RETRACTED

# An Novel Optimization Model for Ideological and Political Course in Colleges under the Environment of BD Mining Technology

**DOI:** 10.1155/2022/1372855

**Published:** 2022-09-06

**Authors:** Xinglin Yang

**Affiliations:** ^1^Department of Philosophy, Nanjing University, Nanjing 210023, China; ^2^The Center for Study of Eco-civilization, Nanjing Forestpolice College, Nanjing 210023, China

## Abstract

The big data (BD) era and pertinent computer science, pedagogy, and educational psychology knowledge are the foundations of this essay, based on the idea of the holistic development of human beings, the IPE (Ideological and Political Education) carrier theory, the new idea of educational development, and the strategy of strengthening the nation through education; the challenges IPECU (Ideological and political education in Colleges and Universities) faces and its path toward optimization are discussed relatively in detail in this paper, which conforms to the context of mega data thinking. The influence of IPECU's subject, object, and educational effect is discussed in this paper, along with tips for how to improve and innovate IPECU in the context of big data. In addition, it is noted that in the age of mega data, we must not only bravely take on challenges, but also actively seize opportunities if we are to realize the innovative and optimized development of IPECU. Moreover, the definitions of mega data and big data prediction function are provided in this paper. IPE can be used with the big data prediction function, which is further explored in this article. In order to realize the innovation of IPE mode in universities, this paper aims to encourage the integration and development of IPE and big data in academic settings.

## 1. Introduction

Our lives now have never-before-seen quantifiable dimensions, and big data is the inspiration behind numerous new products and services [1]. The era of mega data is unquestionably the inevitable wave of network IPE, and big data haVE permeated all aspects of society today. Of course, it goes without saying that objective data are important when analyzing issues [2]. The rapid development of data and informatization in the age of mega data has compelled political thought educators in universities to place a premium on data value and possess corresponding data processing capabilities. Additionally, educational objects are actively thinking and pursuing individuality, which makes the IPE environment in universities more and more complex. Big data is viewed in the context of network IPE as a value concept as opposed to a technical means and tool [3]. A trend that is impossible to ignore is the fusion of education and mega data technology. But the age of mega data also presents a number of difficulties for network IPE, including concerns about data security and privacy. IPECU's carriers exhibit some real-world issues, including a lack of ability to attract college students, a lack of carrier integration, and a lack of ability of traditional carriers to innovate. College students' disinterest in IPE is a result of the practical issues [4]. IPECU's subject and object, as well as all spheres that have an influence on education, are facing previously unheard-of difficulties and challenges. Regardless of the advantages or difficulties that the mega data era brings, network IPE cannot reject and avoid this new environment [5]. As a result, the main focus of current research is on how to apply the big data prediction function to the practical application of IPE, investigate a powerful new application mode, and enhance the impact of IPE.

RETRACTED

IPE must seize the chance presented by the big data era and use data analysis to make life and study more intelligent in the digital information age with big data as the background; To master the personality traits and behavioral norms of the educated, one must cultivate data awareness; mega data information is a powerful tool that can be used to both advance IPE on the Internet and steadily solidify society's dominant ideology [6, 7]. The political thought work should be implemented in universities by political thought educators who are farsighted, take advantage of the opportunities provided by big data technology, and innovate the topic, object, and educational outcome of IPECU. This is because college students are distinctive and unstoppable. IPE information is carried and transmitted by the IPE carrier, and the IPECU and effective IPE carrier cannot be separated from one another [8]. The IPECU carrier aids in information transmission, enhancing the educational process while also assisting the subject and object of instruction, coordinating various educational factors, and providing support. Relevant personnel can transform data into valuable information and forecast the thoughts and actions of educational objects through data mining, analysis, and integration [9]. This is a successful way to resolve IPE's dilemma in the new era of mega data, as well as the outcome of IPE following the trend of the times and seizing the opportunities of science and technology development. Additionally, it offers fresh perspectives for IPE's ecological chain that can lead to revolutionary transformation and long-term sustainability. With regard to IPECU's innovations, this paper discusses the problems it faces and possible paths for improvement in the mega data era:

1. Based on the discipline of IPE itself, this paper makes a preliminary discussion on the challenges faced by IPECU in the era of mega data and its optimization path by comprehensively applying disciplines such as pedagogy, psychology, and computer soft science. It has outstanding characteristics of the times.
2. After defining the concepts related to big data, this paper puts forward new requirements according to the new characteristics of IPECU in the era of mega data, analyzes the challenges faced by IPE, and puts forward the optimization path. At the same time, in the evaluation of IPE, the evaluation effect can be fed back in many directions, and the educational regulation can be carried out in real time. On the basis of this application assumption, the precise customized IPE mode is summarized. The overall thinking is clear and has strong practical significance.

RETRACTED

## 2. Related Work

IPE is an important method and means for the country to carry out mainstream ideological propaganda, improve people's ideological, political, and moral literacy and consciousness, and promote people's free, comprehensive, and sustainable development. How to improve its educational effect is an important topic that experts and scholars have been devoted to.

Zhou believes that political thought educators should analyze the characteristics of mega data and the challenges it brings to IPE, and put forward optimization measures to ensure the standardization, pertinence, effectiveness, and security of online IPE [10]. Wu et al. proposed to explore a new carrier of IPE in order to provide a strong ideological guarantee and spiritual impetus for the development of financial undertakings; therefore, it is proposed to take the leadership, education, management, and activities as the carrier to promote the development of financial undertakings and enhance the penetration of IPE [11]. Wang believes that prediction, as the core function of mega data, has the same characteristics as big data, that is, entity rather than sampling, efficiency rather than accuracy, and correlation rather than causality [12]. Xu et al. believe that in universities, where ideas are active and knowledge is intensive, a great quantity of heterogeneous information data will be generated, which is difficult to be counted and described by the previous traditional methods [9]. Hovdhaugen believes that the application of mega data prediction function in IPE is essentially the inheritance and development of ideological prediction, and is the latest manifestation of ideological prediction under the new background of the mega data era [13, 14]. Che believes that big data should also play a management service function in addition to ideological indoctrination [15]. Ojiako believes that by using big data technology, we can further grasp the essential laws of cognitive development of things from a deeper level based on the mining, analysis, and sorting of massive data, which can be derived and applied to the cultivation field of IPE [16, 17].

RETRACTED

This paper, which is based on the field of IPE itself, provides a preliminary discussion of the difficulties IPECU is facing in the era of mega data and its path to optimization by thoroughly integrating the field's theories of pedagogy, psychology, and computer soft science. The terms “mega data” and “big data prediction function” are defined in this essay. It goes into more detail about how the big data prediction function might be used for IPE. The educational regulation can be implemented in real time while also being fed back into many different directions during the IPE evaluation. The precise customized IPE mode is summarized based on this application presumption.

## 3. Methodology

### 3.1. The Era of Mega Data and Its Characteristics

While thinking about how to better serve all circles, the first task is to clarify its concept and the possibility of its realization [18]. We are in the era of IT, facing the trend of explosive growth of data. The characteristics of sea quantification of data and information require people to have enough data processing ability and more advanced analysis technology [19]. What is “Big Data”? What is the main function of mega data? It is a question that we should consider carefully. There have been many discussions on the concept of mega data in academic circles, but the specific concept of mega data has not yet reached a unified conclusion. Instead, it is constantly changing in the statements of different researchers. Big data is an unprecedented way to obtain valuable products and services or profound insights by analyzing massive data.  Figure 1 shows the characteristics of mega data.

According to the application type of data, big data can be divided into three categories: massive transaction data, massive interactive data, and massive processing data [20]. Massive transaction data mainly refers to the online transaction processing from ERP application to data warehouse application. Massive interactive data mainly comes from the composition of social media data; massive data processing refers to the data-intensive architecture based on the emergence of mega data. Nowadays, before comparing the types and forms of data, it shows diversity characteristics.  Figure 2 shows the operation flow chart of mega data technology.

In this paper, big data is defined as a set of data that cannot be adapted by traditional tools and methods, but can be captured, stored, analyzed, and processed by special sci and tech means, and can gain great value through technical analysis. At the same time, this paper is based on the narrow concept of mega data, focusing on the technology and application of mega data. Big data, in general, is an information asset that requires new tools and models for management and processing. It has the fundamental traits of a huge volume, a wide variety, a low value density, and a high speed. People are now both transmitters and receivers of data due to the ever-evolving growth trend of data resources. Second, the data technology has greatly improved with the development of various hardware data transmission devices like sensors. The rapid development of various advanced transmission devices has made the data more and more effective, and the data is approaching the fundamental properties of things. Mega data prediction function realization has its own operational procedure and realization potential. Because it is supported by a strong theoretical foundation, IPE is distinguished from imagination and fantasy as a field of study by its scientific nature. Mega data currently has a very large scale, it is difficult to collect, manage, and analyze using standard tools, and has a very large monetary value. Massive amounts of data and information can be sorted and analyzed to help people make more informed decisions and update our social practises' values. The obvious benefits of the mega data era are demonstrated by a significant amount of complex information, and the singularity of the mega data era cannot be fully summed up by the sheer volume of data.

RETRACTED

### 3.2. Challenges Faced by IPECU in the Era of Mega Data

For the new development of IPECU, big data opens up new possibilities. We must pay attention to a number of issues that are present in this process, though. Educators currently have limited IT access and a poor understanding of data, which has an impact on the quality of educational materials. The majority of the professors and advisors who teach political thought theory courses at universities have backgrounds in the liberal arts, and as a result, they have very limited skills in processing information from the Internet, big data, and other sources. Throughout the entire teaching process, educators are crucial as mentors and motivators. The big data era will inevitably have an impact on universities' IPE processes if educators cannot adjust to its development. Relying on big data carriers to carry out IPE necessitates that educators possess not only the professional quality and ability of IPE but also the capacity to gather data, perform quantitative analysis, and identify and resolve issues in complex data. There are also some issues with cultivating people in universities given the current state of IPECU. One reason is that the current content of IPECU is not entirely practical, ignoring students' interests and needs and being divorced from the needs of social deviance. As an example, the ideological and moral cultivation and scientific and cultural cultivation have not been completely unified, and problems with college students' low psychological quality, contempt for life under pressure, or high flyers' moral quality, which endanger the society, emerge in endlessly.

RETRACTED

Mega data now plays a significant role in society across all sectors, and some universities have set high standards and made audacious attempts to integrate this technology into IPE's discipline construction. However, this excessive worship of expectations might cause people to reject technology or plunge into the “data-only” concept crisis. That is to say, ignoring or blindly believing in big data is not a good way to increase education's capacity for innovation. Universities are currently investing heavily in hardware technology, and each department has its own customized office application information system software. Information databases are used, but not with enough care; they are separate from one another and do not complement one another. There is still room for improvement in data awareness. Students' information data is vertically and horizontally fragmented, and there is no current summary of the hardware and software data resources within. It is not sufficient for IPECU practise to merely rely on thorough and ideal educational materials and scientifically accurate educational concepts. Additionally, efficient teaching strategies must be offered. The information access of college students is shown in Figure 3.

The extensiveness and complexity of data information sources are determined by the characteristics of mega data, which leads to the ambiguity of information value and the dispersion of high-value information. As a result, some western nations could easily use the Internet to infiltrate ideologies and culture. It is particularly challenging for college students with immature ideas to distinguish authenticity in the face of enormous data, and it is easier to lose oneself in the virtual environment. There are even issues like a lack of social responsibility and hazy moral concept. Money worship, hedonism, and the “universal values” of the West will directly or indirectly affect the educational objects. Additionally, data encryption and the protection of personal information are currently issues with the use of mega data in IPECU. According to the actual situation, there are no laws or regulations related to big data that have been created or supplemented, there is a serious problem with the illegal use of personal information, it is unclear who has the authority to conduct research and what is expected of teachers, and many students violate their privacy by disclosing their personal information. For IPECU and big data technology to work together flawlessly, there is still much work to be done.

RETRACTED

### 3.3. Optimization Path of IPECU in the Era of Mega Data

#### 3.3.1. IPE Should be Targeted and Normative

In educational design, we should play the role of mega data, effectively combine teachers' work experience, grasp students' needs, focus on optimizing students' experience, actively introduce hot cases, carry out targeted classroom seminars, special lectures, social practice and other activities, resolve the problems existing in students' thoughts and behaviors, and strive to achieve the goal pursued by IPE with new teaching materials. Big data can achieve an “accurate portrait” of an individual. If big data is combined with education, educators can use big data technology to analyze students' behavior characteristics and carry out targeted education for them. In the era of mega data, first of all, we should establish and strengthen the awareness of mega data and enhance the sensitivity to data information, which depends on the degree of recognition of the value of data resources and the strong desire to innovate educational methods of political thought educators in universities. The process of ideological and moral formation is shown in Figure 4.

In the big data environment, political thought theory courses in universities shoulder a more important historical mission. Political thought educators need to give new sense of the times in the content and teaching methods of IPE courses, enhance their attraction and influence college students, and expand the main front range of IPE for college students.  Table 1 shows the influence of network information on college students' values.

Students are in a critical period of establishing correct world outlook, outlook on life and values, and they are active in thinking and willing to accept different new things. Their thoughts and behaviors are highly malleable, and they will inevitably be influenced by negative values in the mass information in the era of mega data. Therefore, the process of network IPE should be carried out in a targeted way. Educators should formulate personalized educational contents and methods according to the characteristics of different educational objects, and formulate teaching plans purposefully and hierarchically. At the same time, political thought educators, as instructors and leaders of IPE for students, must further clarify their responsibilities. Political thought educators in universities must keep pace with the times, forge ahead, and constantly improve their educational ability and level in educational practice.

RETRACTED

#### 3.3.2. Improve the Thinking Concept of IPE and Clarify the Boundaries of Mega Data Utilization

In the era of mega data, the network political thought educators not only need a higher level of political theory, but also have the ability to deal with the rapid dissemination of information, which requires educators to effectively master the network technology and network cultural characteristics. Universities should actively build a big data sharing platform that is suitable for IPE, and get rid of the disadvantages of information disconnection among educators and lagging understanding of the ideological changes of educational objects. The analysis of information is a necessary stage from collection to processing, and plays the role of connecting the past with the future. Only through in-depth analysis, can we reveal the internal relationship from scattered data and discover the internal essence of people's thoughts and behaviors. The construction of “big data” in IPE must establish a comprehensive and systematic thinking and a modern information collection system. It is necessary to inherit and carry forward the fine tradition, especially to collect and sort out the data recorded in each historical stage, and to collect all the process data of the current IPE simultaneously, and to mine useful information for analysis. To improve the effectiveness of online IPE, on the one hand, the content of IPE fully reflects the characteristics of real-time data, and changes the traditional static IPE model into a dynamic one. On the other hand, we should broaden the path of IPE on the Internet, innovate educational technology and equipment, and enable the educated people to enjoy learning resources anytime and anywhere. Universities should establish information sharing mechanism to promote the integration of data and information resources among departments. It is an important resource for scientific analysis and inquiry of data. Objective and dynamic data are helpful to understand students' real thoughts, behaviors, values and mental health, help educators fully integrate information resources, carry out creative teaching activities, and promote the effective advancement of IPE science and keep the IPE continuously increasing its effectiveness in the dynamic development of technology. The evaluation of college students' IPE theory course is shown in Figure 5.

RETRACTED

Through the investigation, the current college students' evaluation of the implementation of IPE theory course in our school shows that only 15.16% of them think that teachers can combine resources such as the Internet and have novel education methods.

Mega data awareness, the use of big data technology, a thorough understanding of big data, and a thorough investigation of the legal framework governing the IPE of university faculty and students can all serve as solid assurances and point in the right directions for successfully implementing the IPECU. Big data can quantify the various IPE-related factors and evaluate students in a variety of ways depending on the IPE's emphasis and goals in order to support their social and personal growth. The quantitative relationship between college students' thoughts and behaviors should also be established scientifically. At the same time, a multilevel index evaluation system should be set up, and the index values should be determined using an intelligent big data operation method. By examining the behaviors and habits of the educated objects, network political thought educators can forecast their thoughts and identify potential issues in advance. Faced with the effects of various ideologies and social currents, we should establish and enhance the necessary laws and rules, give management and education attention, and bolster network management and the investigation of false information using technical and legal means. University professors of political thought must understand that while big data can certainly benefit current political thought research in many ways, it is not omnipotent. IPE will eventually lose its true significance in educating people if we attempt to solve all of its problems with data in a blind manner. Therefore, it is essential to standardize the scope of data use, avoid data-only doctrine, and cultivate the big data awareness of political thought educators in universities. Meanwhile, it is essential to improve technical training in pertinent data encryption as well as political thought educators' thinking awareness of data collection from college students. In order to fully exploit its value, student data should not only be used effectively but also reasonably and effectively protected. In order to effectively combine heteronomy and self-discipline to counter inaccurate information, it is also necessary to strengthen netizens' legal awareness, sense of responsibility, and good network moral belief. Finally, it is important to ensure the safety of the educational environment.

## 4. The Application of Mega Data Prediction Function in IPE

IPECU ought to continue due to the mega data era's ongoing advancement trend, follow its development direction, and train IPE students in universities to become talent teams with a thorough understanding of data collection, mining, analysis, and application, as well as the knowledge and skills of professional disciplines. In addition to advancing the IPE along the “calculation” path and enhancing the relevance and accuracy of education, the application of mega data prediction function also strengthens the supervision and regulation of the educational process and guards against the undesirable thoughts and behaviors of the educated objects. The actions and words of college students are frequently captured in their entirety in the age of big data. Through the use of cloud computing, students' ideas and words are transformed into lengthy data codes and stored, leaving a variety of data footprints behind. In order to understand the ideological and behavioral trends of college students for the first time, educators can use big data technology to mine the information traces left by students in daily life, collect, and analyze these information data. If instructors discover that a student has negative tendencies, they can intervene early to stop issues before they start and take the necessary steps to help college students develop in a healthy and constructive way. The first step in the IPE process is creating the plan. Mega data prediction can not only assist educators in predicting the current psychological activity and behavior development trend of all educational objects and individuals, but it can also assist educators in developing sound educational programmes. To better mine the rich feedback data from students, political thought educators in universities should increase their data sensitivity, actively look for relationships between college students' personality traits and their environment and other variables, and have a keen sense of observation. The impact of mega data on college students' lifestyle is depicted in Table 2.

RETRACTED

With the progress and development of data technology, students' communication tools are increasing, and students' communication forms are also very distinctive, so unstructured data information resources will gradually increase. The training of network science and technology knowledge is very necessary for college students to study data IT.

Scientific education program is the link to promote the educational effect to achieve the expected educational purpose. In the process of applying big data prediction function to the design of IPE program, the following steps should be followed:

1. Educators should be good at using big data prediction technology to find problems.
2. Determine the goal of IPE.
3. In the process of making educational programs, we should analyze the characteristics of educational objects through big data.
4. To predict the potential problems of the scheme.
5. Use big data technology to realize the rational allocation of resources.
6. Choose an appropriate education scheme.

Political thought educators can grasp and analyze the prejudgment in time, which makes the IPE management ahead of time and initiative, which is essential for better work. As the last link in the process of IPE, the evaluation stage is not only a judgment of the “curative effect” of staged education, but also a new starting point for improving the educational process, and plays a “baton” role in regulating and optimizing the educational objectives, means, and methods of the next stage. Universities can assist teaching through data analysis, respect the differences of college students, try to push education accurately according to the ideological characteristics and specific needs of educational objects, and explore the quantitative evaluation of educational effects. Make IPE more targeted through quantitative research. The application of mega data in educational evaluation should adhere to the principles of scientificity and operability, the combination of single evaluation and comprehensive evaluation, the combination of micro evaluation and macro evaluation, and the combination of qualitative analysis and quantitative analysis. A perfect educational feedback mechanism can help political thought educators in universities to better understand the attitudes, needs, interests, styles, and other information of each learner in the learning process; and provide them with more targeted learning content or learning suggestions to improve their learning efficiency. The flow chart of the application of mega data and its forecasting function to the daily management of college students is shown in Figure 6.

Through the analysis and processing of a mega data platform, we can investigate the relationship between college students' spiritual lives and their families of origin, lifestyle choices, and interpersonal relationships in order to study the three main viewpoints of contemporary college students as well as their views on the rule of law, morality, consumption, love and marriage, life, etc. Because of the ongoing advancements in mega data prediction technology, it is now possible to use software and algorithms to implement automatic operation and deduction, measure and calculate the thoughts and psychology of educational objects, investigate the fundamental rules governing their behavior, and forecast future development trends. It reduces the amount of work that educators have to do while also promoting “data-driven” decision-making in the educational sector. In order to create an accurate IPE mode, one must rely on big data forecasting technology and create a “personal tailor” IPE mode that adjusts to the unique requirements of the educated object. However, political thought educators in universities should prevent the phenomenon whereby students' freedom of choice is severely constrained by the predicted results or whereby they are forced to act in accordance with the predicted results, thereby robbing them of their freedom of choice.

RETRACTED

## 5. Conclusions

Mega data technology is used in the IPE process to not only further enrich the content of IPECU but also to address a number of current practical issues, enabling IPE to effectively achieve its intended goal of educating people. The meaning and traits of mega data as well as the fundamental traits of information in the mega data era are systematically examined in this essay. On this foundation, it further examines the difficulties IPECU has encountered in the age of mega data and suggests the best course of action for solving the issues. As professors of political thought, they must stay current, closely monitor the pulse of the times, actively think and summarize, and know how to effectively and correctly apply the methods of data mining, data collection, and data processing to IPE. I am hoping that this research can offer IPECU in the new era a theoretical scientific foundation. IPE is a social practise and a sophisticated, systematic project that is evolving as society continues to advance. As a result, I'll keep conducting in-depth research for my upcoming coursework and employment and give IPE my best effort as it grows and innovates.

## Figures and Tables

**Figure 1:** Big data features.

**Figure 2:** Operation flow chart of mega data technology.

**Figure 3:** Ways for college students to obtain information.

**Figure 4:** Formation process of ideological and moral character.

**Figure 5:** College students' evaluation of IPE theory course in our school.

**Figure 6:** Flow chart of application of mega data and its prediction function in college students' daily management.

**Table 1:** The influence of network information on college students' values.

Influence values	Proportion (%)
Great influence, overturning the values of the past	8.76
Great impact, with changes in values in some aspects	50.66
Small impact, will not change their value orientation	40.58

**Table 2:** The influence of mega data on college students' lifestyle.

Lifestyle influence	Proportion (%)
Get the information needed for study and life	82.46
Social patterns change	60.57
Easy to reveal personal privacy information	90.82
It does not matter	1.32

RETRACTED

## Data Availability

The data used to support the findings of this study are available from the author upon request.
